# Synergistic Cytotoxicity between *Elephantopus scaber* and Tamoxifen on MCF-7-Derived Multicellular Tumor Spheroid

**DOI:** 10.1155/2021/6355236

**Published:** 2021-10-19

**Authors:** Wan Yong Ho, Sok Sian Liew, Swee Keong Yeap, Noorjahan Banu Alitheen

**Affiliations:** ^1^Faculty of Science and Engineering, University of Nottingham Malaysia, 43500 Semenyih, Selangor, Malaysia; ^2^China-ASEAN College of Marine Sciences, Xiamen University Malaysia, 43900 Sepang, Selangor, Malaysia; ^3^Faculty of Biotechnology and Biomolecular Sciences, Universiti Putra Malaysia, 43400 Serdang, Selangor, Malaysia

## Abstract

*Elephantopus scaber* Linn, a traditional herb, exhibited anticancer properties, and it was cytotoxic against the monolayer estrogen receptor-positive breast cancer cell line, MCF-7, in the previous study. In order to determine the potential of *E. scaber* as a complementary medicine for breast cancer, this study aimed to evaluate the synergism between *E. scaber* and tamoxifen in cytotoxicity using MCF-7 in the form of 3-dimensional multicellular tumor spheroid (MCTS) cultures. MCTS represents a more reliable model for studying drug penetration as compared to monolayer cells due to its greater resemblance to solid tumor. Combination of *E. scaber* ethanol extract and tamoxifen, which were used in concentrations lower than their respective IC_50_ values, had successfully induced apoptosis on MCTS in this study. The combinatorial treatment showed >58% increase of lactate dehydrogenase release in cell media, cell cycle arrest at the S phase, and 1.3 fold increase in depolarization of mitochondrial membrane potential. The treated MCTS also experienced DNA fragmentation; this had been quantified by TUNEL-positive assay, which showed >64% increase in DNA damaged cells. Higher externalization of phospatidylserine and distorted and disintegrated spheroids stained by acridine orange/propidium iodide showed that the cell death was mainly due to apoptosis. Further exploration showed that the combinatorial treatment elevated caspases-8 and 9 activities involving both extrinsic and intrinsic pathways of apoptosis. The treatment also upregulated the expression of proapoptotic gene HSP 105 and downregulated the expression of prosurvival genes such as c-Jun, ICAM1, and VEGF. In conclusion, these results suggested that the coupling of *E. scaber* to low concentration of tamoxifen showed synergism in cytotoxicity and reducing drug resistance in estrogen receptor-positive breast cancer.

## 1. Introduction

Female breast cancer is the most diagnosed cancer worldwide, and it accounts for 1 in every 6 cancer deaths in year 2020 [1]. Hormonal therapy is one of the most common treatments in breast cancer. It is effective towards majority of the breast carcinomas that express significant levels of estrogen receptor [2]. Tamoxifen—the oldest and the most prescribed drug in breast cancer hormonal therapy—blocks estradiol from binding to the malignant cells and inhibits the growth of estrogen receptor-positive breast cancer cells. Despite treatment advancement, the use of modern drugs for breast cancer treatment is still associated with a variety of health and psychological problems [3,4]. Therefore, folk medicinal herb has been applied as complementary and alternative medicine alongside modern therapeutics to many cancer patients [5]. It enhances the tolerance of patients to radiotherapy, increases the sensitization of cancer cells to chemotherapy, and reduces the side effects from cancer treatment [6].

Growing resistance to cancer cells with single treatment also promotes the use of multiple drugs or therapeutic remedies with different mechanisms of action for synergistic effect against cancer [7]. For instance, herbs such as *Vernonia amygdalina* [8] and flaxseed [9] have been shown to augment the drug cytotoxic effect on MCF-7 breast cancer cells with reduced drug dosage. *Elephantopus scaber* Linn (also called as Elephant's foot) is a perennial herb from the Asteraceae family that grows in many tropical countries. The whole plant of this herb and its extracts can be consumed for diverse traditional treatment. This plant extract and the isolated compound have showed antiproliferative activities towards many cancer cell lines from the lung, nasopharyngeal, colon, and liver [10–13]. Our previous study used monolayer MCF-7 cells model to show the strongest cytotoxic effect exhibited by the ethanol extract of *E. scaber* than other types of extracts, suggesting that the extract may be a potential candidate in herb-drug treatment for estrogen receptor-positive breast cancer [14]. However, the interaction of *E. scaber* with breast cancer drug had not been reported in any literature to date.

In our previous study, we have identified a high-throughput screening using 3-dimensional multicellular tumor spheroid (MCTS) derived from MCF-7, and the MCTS responded well to tamoxifen after 4 days of exposure [15]. MCTS presents a more reliable *in vitro* model that resembles highly to a solid tumor, recreates hypoxic tumor environment, and bridges the knowledge gap between *in vitro* monolayer cancer cell and *in vivo* tumor [16]. This study aimed to evaluate synergism between *E. scaber* and tamoxifen in cytotoxicity on MCTS cultures of MCF-7. We hypothesized that the combination of *E. scaber* and tamoxifen would trigger greater apoptosis in the MCTS cultures of MCF-7 by activating proapoptotic genes and proteins while inhibiting prosurvival genes.

## 2. Materials and Methods

### 2.1. Preparation of *E. scaber* Ethanol Extract

*E. scaber* used in this work was collected from Georgetown, Penang. The plant was identified and deposited with voucher specimen number FRI65693 in the Forest Research Institute Malaysia (FRIM), Kepong, Selangor. Ethanolic leaf extract of *E. scaber* was prepared as described previously [14]. Briefly, the leaves of *E. scaber* were powdered and subjected to extraction for three times using absolute ethanol at room temperature. All the content of each extraction was mixed and filtered through grade 1 Whatman filter paper. The filtrate was then evaporated to dry under reduced pressure at <40°C using Aspirator A-3S (EYELA, Japan). We obtained a final yield of 8% of the dried leaves initial weight, and this ethanol extract was stored at −20°C until use.

### 2.2. Cell Culture

The estrogen-dependent human breast adenocarcinoma, MCF-7, was obtained from American Type Culture Collection (ATCC, USA). The cells were maintained in Dulbecco's modified eagle medium (DMEM) (Sigma, USA) supplemented with 10% (v/v) of heat-inactivated foetal bovine serum (FBS) (PAA, Austria), 100 I.U./ml penicillin, and 100 ng/ml streptomycin (PAA, Austria). The cells were cultured at 37°C in a 90% humidified incubator with 5% CO_2_.

### 2.3. MTT Cytotoxic Assay

Various concentrations of *E. scaber* (20, 40, 60, 80, and 100 *μ*g/mL) were added as treatment, either with or without the combination with a few concentrations of tamoxifen citrate at 1.56, 3.125, or 6.25 *μ*g/mL, respectively, for a total of 4 days. Tamoxifen citrate contains active ingredient tamoxifen, and it is mentioned as tamoxifen below. Subsequently, 3-(4,5-dimethylthiazol-2-yl)-2,5-diphenyl tetrazolium bromide (MTT) assay and the generation of MCTS cultures were carried out according to the methods described previously [15]. Briefly, after 4 days of treatment, 20 *μ*l of MTT solution was added into each well containing the MCTS cultures and incubated for 4 hours. The treated MCTS cultures were transferred to new, flat bottom 96-well plate and centrifuged at 1,000 × g for 5 minutes. Then, 150 *μ*l of media was aspirated from each well, and the plate was blot dried on paper towels, followed by adding 100 *μ*l of DMSO into each well. Finally, absorbance was recorded at 570 nm using the *μ*Quant enzyme-linked immunosorbent assay (ELISA) Reader (Bio-tek Instruments, USA). The concentrations of tamoxifen, *E. scaber*, and combination treatment that resulted in 50% of cell death (IC_50_) were determined from respective dose-response curves. Synergistic effects of *E. scaber* and tamoxifen were measured by calculating combination index (CI) and dose reduction index (DRI) values using CompuSyn (ComboSyn lnc, US). CI < 1, =1, and >1 indicates synergistic, additive, and antagonistic effect of the combination.

### 2.4. Cell Seeding, Treatment, and Dissociation

MCTS cultures were cultured according to the methods described previously [15]. For all the assays from Section 2.5to 2.12, the cultures were subjected to five groups of treatment, namely ES60 (60 *μ*g/mL *E. scaber*), ES60 + TC3 (60 *μ*g/mL *E. scaber* with 3.125 *μ*g/mL of tamoxifen), ES60 + TC6 (60 vg/mL *E. scaber* with 6.25 *μ*g/mL of tamoxifen), TC3 (3.125 *μ*g/mL of tamoxifen), and TC6 (6.25 *μ*g/mL of tamoxifen) for a total of four days. One group was left untreated to serve as the negative control. MCTS cultures were subjected to enzymatic dissociation into single cell suspension before being assayed for following activities in Section 2.8to 2.11: cell cycle analysis, mitochondrial membrane potential (ΔΨm) detection, terminal dUTP Nick End Labeling (TUNEL) assay, and caspase-8 and caspase-9 fluorometric activity assay. Briefly, the cultures went through washing twice in 1 ml of PBS-BSA-EDTA solution followed by incubating in 500 *μ*l of Accutase™ solution (PAA, Austria) at 37°C for 20 minutes to allow cells dissociating completely. The cells were then centrifuged at 300 × g for 5 minutes followed by washing twice with PBS-BSA-EDTA solution.

### 2.5. CytoTox 96® Nonradioactive Cytotoxicity Assay

Cytotoxicity of the treatment was also assessed using the CytoTox 96® Non-Radioactive cytotoxicity assay (Promega, USA) according to the manufacturer's instructions. Release of lactate dehydrogenase (LDH) into culture medium was measured after 4 days of treatment. Firstly, 20 *μ*l of 10x lysis solution was added into half of the untreated wells prior to assay to induce maximum LDH release. After 45 minutes, the plate was centrifuged at 300 × g for 4 minutes, and 50 *μ*L of supernatant from each well was transferred to a new plate. Subsequently, 50 *μ*l of TMB substrate was added into each well, and the plate was incubated at room temperature for 30 minutes in the dark. Next, 50 *μ*l of stop solution was added into each well and the absorbance was measured at 492 nm using the µ Quant ELISA Reader (Bio-tek Instruments, USA). Percentage of cytotoxicity was calculated according to

(1) $$\begin{array}{c} \text{percentage of cytotoxicity}=\frac{\text{experimental sample absorbance}}{\text{maximum release absorabnce}}\times 100. \end{array}$$

### 2.6. Flow Cytometric Detection of Apoptosis by Annexin V and Propidium Iodide Staining

MCTS cultures were stained by annexin V-FITC and propidium iodide according to the manufacturer's protocol (Becton Dickinson, USA). Phosphatidylserine externalization was assessed by quantifying surface annexin V-FITC and propidium iodide using FACS Calibur flow cytometer. The analysis was performed as previously described [14].

### 2.7. Fluorescent Microscopic Assessment of Apoptosis by Acridine Orange and Propidium Iodide Staining

Apoptosis assessment of MCTS cultures using acridine orange and propidium iodide double staining was carried out according to the method described previously [14]. The staining dye (10 *μ*g/ml of acridine orange and propidium iodide each) was added into MCTS cultures and 10 *μ*l of the stained cells were observed under an inverted fluorescent microscope (Nikon, Japan).

### 2.8. Cell Cycle Analysis

Cell cycle analysis of MCTS cultures was carried out with the FACS Calibur flow cytometer according to the manufacturer's protocol (Becton Dickinson, USA). In brief, cells were harvested, washed in PBS, and treated with RNAse and Triton-X. The cells were then subjected to flow cytometer analysis.

### 2.9. Flow Cytometry Mitochondrial Membrane Potential (ΔΨm) Detection

Depolarization of mitochondria was detected using the BD™ MitoScreen Kit (Becton Dickinson, USA), following manufacturer's instruction. Cells were harvested and incubated with JC-1 (5,5′,6,6′-tetrachloro-1,1′,3,3′-tetraethylbenzimidazolcarbocyanine iodide, a lipophilic fluorochrome) working solution made from dilution of JC-1 stock solution and assay buffer at 1 : 100 ratio. After incubating the mixture at 37°C for 15 minutes, the cells were washed with assay buffer twice and proceeded to FACS analysis.

### 2.10. Terminal dUTP Nick End Labeling (TUNEL) Assay

TUNEL assay was carried out according to the protocol of the APO-DIRECT™ Kit (Becton Dickinson, USA). In brief, the cell suspension was stained and subjected to analysis using FACS Calibur flow cytometer as previously described [14].

### 2.11. Caspase-8 and Caspase-9 Fluorometric Activity Assay

The activities of caspase-8 and caspase-9 were determined by detecting cleavage of substrates specific for caspase-8 (IETD-AFC) and caspase-9 (LEHD-AFC). Colorimetric measurements were carried out according to the protocol of the FLICE/Caspase-8 Colorimetric Assay Kit (BioVision, Inc., USA) and Caspase-9 Colorimetric Assay Kit (BioVision, Inc., USA).

### 2.12. mRNA Expression Analysis

#### 2.12.1. Total RNA Purification from MCTS Culture

Total RNA extraction was performed using the MasterPure RNA Purification kit (Epicentre Technologies, USA) according to the manufacturer's protocol. First, cell pellet that contained 1 × 10^6^ cells was resuspended into 300 *μ*L of Tissue and Cell Lysis Solution (that contained 50 *μ*g of Proteinase K) and incubated at 65°C for 15 minutes with intermittent mixing every 5 minutes. Then, the mixture was transferred to ice for 5 minutes, followed by the addition of 175 *μ*L of MPC Protein Precipitation Reagent. The cell suspension was mixed vigorously before centrifuged at 12,000 × g for 10 minutes at 4°C. The recovered supernatant was transferred to 500 *μ*L of isopropanol and inverted for mixing thoroughly. Nucleic acids were precipitated by centrifugation at 12,000 × g for 10 minutes at 4°C. After that, isopropanol was removed carefully from the tube, and the nucleic acids were subjected to DNA removal by incubation with 5 U of DNase I at 37°C for 30 minutes. Upon completion, the solution was added with 200 *μ*L of *T* and C Lysis Solution and 200 *μ*L of MPC Protein Precipitation Reagent and further incubated on ice for 5 minutes. Residual protein in the mixture was removed by centrifugation at 12,000 × g for 10 minutes at 4°C. Total RNA in the recovered supernatant was then precipitated once more using 500 *μ*L of isopropanol. Then, the mixture was centrifuged again at 12,000 × g for 10 minutes at 4°C. After washing twice in 70% ethanol, total RNA pellet was resuspended in 30 *μ*L of RNase-free water. Following this, the quality and concentration of the RNA samples were determined using NanoPhotometer (Impend, Germany), while integrity of the RNA samples was analysed using the 1% TAE agarose gel electrophoresis. Validation of RNA integrity as well as purity prior to usage in downstream qRT-PCR application is crucial to provide more accurate and reliable results. OD_260/280_ ratios greater than 1.8 are an indication that a given RNA sample is free of protein contamination, while OD_260/230_ ratios of more than 2.0 imply that the sample is free of phenolic or polysaccharide contamination [17]. Generally, 28S rRNA and 18S rRNA bands that showed a ratio of 2 : 1 were considered as of high quality. However, Imbeaud et al. also showed that any RNA band that displayed a 28S rRNA : 18S rRNA ratio of more than 1 could also be considered as of good quality [18].

### 2.13. First Strand Synthesis

Synthesis of cDNA from the purified total RNA was carried out according to manufacturer's instruction of the QuantiTect® Reverse Transcription kit (Qiagen, USA). RNA samples of high quality with *A*_260/280_ ratios between 1.8 and 2.0 and *A*_260/230_ ratios more than 2.2 were used for first strand synthesis. In brief, 1 *μ*g of RNA sample was first added with 2 *μ*L of 7x gDNA Wipeout Buffer. The volume was then adjusted to 14 *μ*L using RNase-free water, and the mixture was incubated at 42°C for 2 minutes, followed by cooling on ice immediately. A reverse transcription reaction mixture was prepared by mixing 1 *μ*L of Quantiscript Reverse Transcriptase, 4 *μ*L of 5x Quantiscript RT buffer, and 1 *μ*L of RT Primer Mix. This reaction mixture was then added to the template RNA mixture and subjected to incubation at 42°C for 15 minutes in the Multigene thermocycler (Labnet International, USA). A final incubation for 3 minutes at 95°C was carried out to inactivate the Quantiscript Reverse Transcriptase. The cDNA products were then cooled down to 4°C and kept at −20°C prior to use.

### 2.14. Primer Design

The primer pairs for housekeeping genes and genes of interest were designed using the Primer Premier 5 software (PREMIER Biosoft Int., USA). Primers were selected to bind specifically to human cDNA using the primer-BLAST program (http://www.ncbi.nlm.nih.gov/tools/primer-blast). Sequences, properties, and GenBank Accession numbers of the primers are listed in Table 1.

### 2.15. Quantitative Real-Time PCR

Relative expression of the target genes (c-Jun, heat shock protein (HSP) 105, intercellular adhesion molecule (ICAM)-1, and vascular endothelial growth factor (VEGF)) and the endogenous controls (Table 1) were determined using QuantiFast® SYBR® Green PCR kit (Qiagen, USA) according to the manufacturer's instruction. Real-time reaction mixture was prepared by mixing 10 *μ*L of 2x QuantiFast SYBR Green PCR master mix, 0.3 *μ*M of each primer, 50 ng of template cDNA, and RNase-free water to a total volume of 20 *μ*L. The reactions were carried out in 96-well plates using the iQ5 multi-colour Real-time Detection System (Bio-Rad Laboratories, Inc. USA). Thermal cycling was initiated at 95°C for 10 minutes, followed by 40 cycles consisting of denaturation at 95°C for 10 seconds and combined annealing/extension steps at 60°C (for 18S rRNA, *β*-actin, HSP 105, ICAM1, and VEGF) or 55°C (for GAPDH and c-Jun). Following the completion of PCR amplification, a melting curve analysis was performed by slowly heating the samples from 55°C to 95°C at 0.2°C/s, while the fluorescence was measured continuously. GAPDH, *β*-actin, and 18s rRNA were used as the reference genes for internal control. The endogenous genes amplification of the control cDNA sample was carried out on every plate to provide internal control marker for comparison of the samples that were run at different times on different plates.

Data analysis was performed according to the relative quantification using the 2^−ΔΔCT^ method [19]. The 2^−ΔΔCT^ method quantifies changes in target gene expression relative to the reference group used, such as the untreated control in this study. In order to perform the 2^−ΔΔCT^ method, efficiencies of the target and reference genes should be approximately equal and close to 100% in the exponential phase of PCR [19]. Therefore, a standard curve was established for each target and the endogenous control to facilitate the calculation of PCR efficiency. A relative standard curve of target and reference gene for quantification of qRT-PCR product was generated by dilution of cDNA from the calibrator (untreated control). The PCR efficiencies of all the target and endogenous genes used in this study were in the range of 100 ± 10%. Gene expression of each sample was represented by the threshold cycle (*C*_*T*_) value, which was defined as the cycle number of which sample fluorescence exceeds a chosen threshold above background fluorescence [20]. The relative stability of the three reference genes was calculated using geNORM analysis before *C*_*T*_ value of each target gene was normalized to the reference genes. The relative quantification of each sample was then calculated using Equation (2).

(2) $$\begin{array}{c} \text{Comparative expression level}=2^{-\Delta \Delta C_{T}},\\ \Delta \Delta C_{T}=\Delta C_{T}\;\left(\text{treated sample}\right)-\Delta C_{T}\;\left(\text{untreated sample}\right),\\ \Delta C_{T}\;\left(\text{treated sample}\right)=C_{T}{\left(\text{target}\right)}_{\text{treated}}-C_{T}\;{\left(\text{endogenous reference}\right)}_{\text{treated}},\\ \Delta C_{T}\;\left(\text{untreated sample}\right)=C_{T}{\left(\text{target}\right)}_{\text{untreated}}-C_{T}\;{\left(\text{endogenous reference}\right)}_{\text{untreated}}. \end{array}$$

### 2.16. Statistical Analysis

The experiments were tested in three independent experiments and each independent experiments with three technical replicates. The results were expressed as mean ± standard error on the mean (SEM). Difference between means was evaluated using the ANOVA test (one way) followed by the Duncan test, and *p* ≤ 0.05 was taken as statistically significant.

## 3. Results

### 3.1. Cytotoxicity Evaluation of *E. scaber*, Tamoxifen, and Their Combinatorial Treatment against Multicellular Tumor Spheroidal (MCTS) Cultures of MCF-7

MTT assay was carried out to evaluate the cell viability of MCTS cultures after four days of treatment. The results showed that the IC_50_ value of *E. scaber* ethanol extract was 101.33 *μ*g/mL. Our previous study has shown that IC_50_ value of tamoxifen was 12.67 *μ*g/mL [15]. Various combinations of the extract and tamoxifen at concentrations lower than their respective IC_50_ values were tested, and the result (Figure 1) showed synergism of combinatorial treatment at most of the concentrations tested. The cell viability between treatments with *E. scaber* alone and when coupled with 1.56 *μ*g/mL of tamoxifen did not differ much. However, when 3.125 *μ*g/mL and 6.25 *μ*g/mL of tamoxifen were used, respectively, in combination with *E. scaber*, cell viability was significantly lowered compared to treatment with the extract alone with the combination index (CI) values 0.886 and 0.73, respectively. Although 6.25 *μ*g/mL of tamoxifen showed better cytotoxic effect than of 3.125 *μ*g/mL, both concentrations showed a more drastic drop in cell viability—approximately 50% of cell death—when 60 *μ*g/mL *E. scaber* was applied. The dose reduction index (DRI) values showed that IC_50_ dose of tamoxifen at 3.125 *μ*g/mL and 6.25 vg/mL could be reduced up to 2.46 fold and 3.66 fold, respectively, when they were used in combination with 60 *μ*g/mL *E. scaber* ethanol extract. Hence, these two combinatorial treatments (60 *μ*g/mL *E. scaber* with 3.125 vg/mL tamoxifen and 60 *μ*g/mL *E. scaber* with 6.25 *μ*g/mL tamoxifen) were selected for downstream synergistic studies between *E. scaber* ethanol extract and tamoxifen on MCF-7 MCTS cultures.

### 3.2. Assessment of Lactate Dehydrogenase (LDH) Release by MCF-7 MCTS Cultures Treated with *E. scaber*, Tamoxifen, and Their Combinatorial Treatment

Cellular membrane damage releases lactate dehydrogenase (LDH), and this can be quantified to compare the level of cytotoxicity among treatments. The results in Figure 2 showed that untreated MCTS (negative control group) secreted a basal amount of LDH, about 36.59 ± 0.03% of maximum LDH content. Treatment with 60 *μ*g/mL *E. scaber* and 3.125 *μ*g/mL of tamoxifen (ES60 + TC3) induced LDH release of 94.78 ± 0.08%, while treatment with 60 *μ*g/mL *E. scaber* and 6.25 *μ*g/mL of tamoxifen (ES60 + TC6) induced 97.58 ± 0.02%. The level of cytotoxicity in both combination groups was higher than the individual treatment with ES60, TC3, and TC6, proving synergism of the herb-drug treatment.

### 3.3. Induction of Apoptosis in MCF-7 MCTS Cultures by Herb-Drug Combinatorial Treatment in Comparison to Single Dosage of *E. Scaber* and Tamoxifen

Phosphatidylserine externalization is an early event during apoptosis; it was assessed here via annexin V (bound phoshatidylserine) and propidium iodide (vital dye) staining with flow cytometry to detect whether the induction of cell death associated with apoptosis or necrosis quantitatively [21]. Both the treatments with TC3 and TC6 increased the population of cells with externalized phosphatidylserine in comparison to the control group, but the apoptotic effect by the latter was greater (Figure 3). Treatment with ES60 increased phosphatidylserine externalization, whereby 27.01 ± 0.62% of cells remained excluded from propidium iodide (indicated early apoptosis), while 33.07 ± 3.85% of cells were stained with propidium iodide (indicated late apoptosis). Combinatorial treatment with ES60 + TC3 and ES60 + TC6 significantly increased early apoptosis event to 33.49 ± 0.02% and 42.88 ± 3.42%, respectively. In contrast with increasing cell population into early apoptosis, combinatorial treatment facilitated cells into late apoptosis slightly more than the treatment with TC3, TC6 alone, but to a percentage that is similar to that of treatment with the herb alone (ES60).

### 3.4. Fluorescent Microscopy Assessment of MCF-7 MCTS Cultures Treated by *E. Scaber*, Tamoxifen, and Their Combinatorial Treatment

Morphological features of the whole solid structure of MCTS cultures were assessed under fluorescent microscopy after double staining with the fluorescent dyes—acridine orange and propidium iodide. The untreated control in Figure 4(a) showed a compact three-dimensional spheroidal culture with much viable cells inside the culture and surrounded by a thin layer of viable cells (stained green by acridine orange). Outer layer of spheroid became thinner with an increase of apoptotic and necrotic cells (stained orange and red with propidium iodide) after incubation with ES60 (Figure 4(b)), TC3 (Figure 4(c)), and TC6 (Figure 4(d)) for 4 days. Treatment with each ES60 and TC6 disintegrated cells from the three-dimensional solid structure. Combinatorial treatment with ES60 + TC3 (Figure 4(e)) and ES60 + TC6 (Figure 4(f)) distorted organization of spheroids to a greater extend compared to single treatment: thinning of the outer layer extended to thinning of the whole solid structure, more cells disintegrated, cultures shrunk in size, greater apoptosis, and necrosis observed. This further supported the synergism between *E. scaber* and tamoxifen on MCF-7 MCTS cultures.

Cells that are stained green indicate viable cells; cells that are stained orange or yellow-red (orange arrows) represent apoptotic cells, while cells that are stained red indicate necrotic cells (magnification: 40x, scale bar: 200 *μ*m).

### 3.5. Effect of *E. scaber*, Tamoxifen, and Their Combinatorial Treatment on Cell Cycle Progression of MCF-7 MCTS Culture

Cell cycle progression of MCF-7 cells in the MCTS culture was examined using flow cytometer (Figure 5). Under standard conditions, most of the MCF-7 cells (71.35 ± 1.38%) in the control group were in quiescence the G0/G1 phase; 13.57 ± 0.76% of cells in the S phase; 15.07 ± 0.86% of cells in the G2 + M phase. Majority of the cells in both TC3 (72.19 ± 1.31%) and TC6 (72.85 ± 1.49%) groups also remained in the G0/G1 phase, at percentages slightly higher than the control group, but the difference was not statistically significant. However, accumulation of cells in the G0/G1 phase declined significantly to 52.89 ± 0.64% in the ES60 + TC3 group and 50.81 ± 0.20% in the ES60 + TC6 group. Treatment with ES60 alone has significantly decreased cells in the G0/G1 phase (50.48 ± 1.24%), increased cells at the S phase (28.65 ± 1.94%), and moderately increased cells at the G2 + M phase compared to the control culture. Although treatment with TC3 and TC6 did not increase cells in the S phase, the addition of ES60 to the tamoxifen treatment increased the accumulation of cells in the S phase significantly to 28.99 ± 1.54% (ES60 + TC3) and 30.49 ± 1.84% (ES60 + TC6); this suggested effect of ES60 at the S phase cell cycle arrest in combinatorial treatment.

### 3.6. Effect of *E. scaber*, Tamoxifen, and Their Combinatorial Treatment on the Alterations of Mitochondrial Membrane Potential in MCF-7 MCTS Cultures

Mitochondrial membrane potential (ΔΨm) of MCTS cultures was evaluated by monitoring the uptake of JC-1 and formation of J-aggregates using flow cytometer (Figure 6). Depolarization in ΔΨm of the spheroid culture from treatment groups was normalized to the control group for direct comparison. Upon treatment with *E. scaber* ethanol extract and tamoxifen, ΔΨm of the MCTS cultures depolarized and JC-1 aggregated, as shown by increased orange-red fluorescence. Treatment with ES60 increased the depolarization to 1.26 fold, while both the treatment with TC3 and TC6 increased the depolarization to 1.21 fold. Synergism of combinatorial treatment was also observed where ES60 + TC3 and ES60 + TC6 further promoted the depolarization of ΔΨm to 1.30 fold and 1.36 fold, respectively.

### 3.7. *E. scaber* Enhanced DNA Fragmentation in MCF-7 MCTS Cultures When Added to Tamoxifen Treatment in Comparison to Induction by Tamoxifen Alone

In addition to qualitative visualization for DNA fragmentation, TUNEL assay incorporated labelled deoxyuridine at sites of DNA breaks and measured DNA fragmentation quantitatively using flow cytometer. A total of 8.44 ± 0.23% of the cells in MCTS cultures from the control group underwent DNA fragmentation after 4 days of incubation (Figure 7). All treatment increased TUNEL-positive cells significantly compared to the control. Treatment with ES60 markedly increased TUNEL-positive cells to 62.80 ± 0.37% in comparison to the treatment with TC3 or TC6, which showed only 20.29 ± 1.64% and 28.21 ± 0.42% of TUNEL-positive cells, respectively. Both herb-drug groups showed synergism in promoting DNA fragmentation: 72.44 ± 0.23% of TUNEL-positive cells in treatment with ES60 + TC3 and treatment with ES60 + TC6 further increased the TUNEL-positive cells to 74.31 ± 0.64%.

### 3.8. Regulation of Caspases 8 and 9 Activities in MCF-7 MCTS Cultures by *E. scaber*, Tamoxifen, and Their Combinatorial Treatment

The regulation of caspase-8 and caspase-9 activities was determined using a colorimetric assay. Activities of the caspases in the control group were adjusted to the value of 1 unit; the other groups values were normalized to the control value and presented as fold change in comparison to the control. Both activities of caspase-8 and caspase-9 (Figure 8) increased but not statistically significant compared to control after 4 days for all treatment. Caspase-8 activity was slightly increased to 1.04 fold after treatment with TC3 and to 1.05 fold after treatment with TC6. Treatment with ES60 caused higher caspase-8 activity with 1.14 fold increase; however, treatment with both ES60 + TC3 and ES60 + TC6 appeared to slightly reduce caspase-8 activity when compared to treatment with ES60 alone. Caspase-9 activity was elevated in treatment with TC3 (1.03 fold), TC6 (1.04 fold), and the highest was recorded with ES60 at 1.09 fold. Although treatment with ES60 + TC3 only induced caspase-9 activity to 1.08 fold (slightly lower than that of ES60), the activity was elevated to 1.11 fold when a higher drug concentration (TC6) was used together with ES60.

### 3.9. Evaluation of the Expression of Several Apoptosis-Related Genes in MCF-7 MCTS Cultures by Real-Time PCR

mRNA expressions of c-Jun (Figure 9), HSP 105 (Figure 10), ICAM1 (Figure 11), and VEGF-A (Figure 12) were studied using the quantitative real-time PCR assay. The untreated control group has its mRNA expressions adjusted to the value of 1 unit; other groups values were normalized to this control value and presented as fold change compared to the control. The mRNA expressions of all 4 genes were upregulated in proportion to increased concentration of tamoxifen. Treatment with TC3 induced 1.12 fold, 2.11 fold, 1.07 fold, and 1.11 fold, while treatment with TC6 further elevated to 2.41 fold, 3.65 fold, 2.13 fold, and 2.13 fold for c-Jun, HSP 105, ICAM1, and VEGF-A mRNA expression, respectively. In contrast, only upregulation of HSP 105 (4.99 fold) was observed after 4-day exposure to ES60. The expressions of c-Jun, ICAM1, and VEGF-A reduced significantly to 0.60 fold, 0.27 fold, and 0.44 fold, respectively, after exposure to ES60. Treatment with ES60 + TC3 and ES60 + TC6 also reduced mRNA expression of these three genes in dosage-dependent manner for two of the following genes. Combinatorial treatment of ES60 + TC3 reduced the expression of c-Jun and VEGF to 0.60 fold and 0.32 fold, while ES60 + TC6 further reduced the expression to 0.38 fold and 0.20 fold, respectively. However, the downregulation of ICAM1 expression was more significant in the ES60 + TC3 (0.28 fold) than in ES60 + TC6 (0.51 fold). For HSP 105, ES60 + TC3 was capable to increase the expression remarkably to 17.68 fold, while ES60 + TC6 increased the expression to just 1.53 fold.

## 4. Discussion

*E. scaber* ethanol extract successfully enhanced cytotoxicity of tamoxifen against estrogen-dependent breast cancer cells in this study. The combinatorial treatment was effective showing synergism between herb and drug; this could serve as the first evidence to promote the use of *E. scaber* in herb-drug treatment for breast cancer with lower drug concentration to reduce drug resistance. Subsequent assays of *E. scaber* and the combinatorial treatment revealed signs of apoptosis and players involved in cell death. ES60 could stimulate 50% cell death with the addition of tamoxifen at concentrations as low as 3.125 *μ*g/mL and 6.25 *μ*g/mL, as shown by the MTT assay (Figure 1) and elevation of LDH release into culture medium (Figure 2). Phosphatidylserine externalization analysis (Figure 3) and acridine orange/propidium iodide staining (Figure 4) indicated that treatment with ES60 + TC3 and ES60 + TC6 induced cell death via apoptosis.

Treatment with ES60 arrested the cells mostly at the S phase before rendered to cell death (Figure 5). Treatment with TC3 and TC6 resulted in growth arrest in the G0/G1 phase although the difference was not statistically significant. It is well understood that antiestrogen drug, tamoxifen, inhibits the growth of estrogen-dependent breast cancer cell via G1 cell cycle arrest; however, recent studies reported other signaling pathways contributing to its apoptotic effect [21,22]. Cyclin-dependent kinases govern cell cycle progression and are able to halt the cell cycle at certain checkpoints. Their activities can be regulated by cyclin binding or by inhibiting of kinase inhibitors such as p21^CIP1^ and p27^KIP1^. Promotion of both p21^CIP1^ and p27^KIP1^ is associated with cell cycle arrest in the G0/G1 and S phases [23]. However, only p27^KIP1^ is responsible for regulating cell cycle arrest through the S phase under certain circumstances such as hypoxia [24]. It is postulated that increased level of p27^KIP1^ by *E. scaber* could be essential for inducing the S phase arrest in the MCTS cultures, while elevated level of p21^CIP1^ by tamoxifen might be more vital for executing the G0/G1 phase arrest. In this study, ES60 + TC3 and ES60 + TC6 resulted in the S phase arrest that was similar to ES60. Hence, it was apparent that the influence of *E. scaber* was more prominent than tamoxifen in regulating cell cycle progression when the two were used concomitantly.

Combinatorial treatment and treatment with ES60 alone triggered more severe DNA fragmentation in the MCTS cultures compared to low concentrations of tamoxifen as shown in TUNEL assay (Figure 7). DNA damage detected by sensor protein directs cells for cell cycle arrest, apoptosis, damage-induced transcription, and DNA repair via DNA-damage response pathway [25]. Both S phase cell cycle arrest and DNA fragmentation contributed by ES60 were able to induce apoptosis in MCTS cultures.

In order to determine underlying mechanism of *E. scaber* in inducing apoptosis, we also examined mitochondrial activities via MTT assay (Figure 1) and depolarization of mitochondrial potential (Figure 6) in treated MCTS cultures. Apoptosis can take place through intrinsic pathway that involves caspase-9 and extrinsic pathway that involves caspase-8. Both caspases-9 and 8 act as initiator caspases that activate downstream effector caspases to propagate death signals. Caspase-9 is activated when mitochondrial membrane disrupts, while caspase-8 is activated after a series of events upon binding to death receptor-associated proteins [24, 25]. Elevated caspase-9 activity (Figure 8) supported the activation of mitochondrial-dependent apoptosis in the MCTS cultures by *E. scaber,* tamoxifen, as well as their combinatorial treatment. In combinatorial treatment, caspase-8 activity declined proportionally with increasing concentration of tamoxifen, while caspase-9 showed in reverse (Figure 8). Cytotoxic effect of the herb-drug treatment was probably contributed more by caspase-9 activation than caspase-8 activation, suggesting that the herb-drug treatment was mitochondrial dependent.

A few key gene expressions studied here explained some underlying mechanism of *E. scaber* in inducing apoptosis. HSP 105 is a molecular chaperone localized in the cytoplasm of human cells; its mRNA expression can be induced in response to a variety of stress stimuli, including heat shock, oxidative stress, and chemical stress [26]. Significant upregulated mRNA expression of HSP 105 (Figure 10) indicated that both *E. scaber* and tamoxifen generated stress in the MCTS cultures. ES60 + TC3 treatment markedly increased the expression of HSP105, while the combination of ES60 + TC6 decreased its mRNA expression when compared to individual treatment of ES60 and TC6 (Figure 10). This effect maybe contributed by the specific regulation of HSP105 induction by the ES60 + TC3, which showed better synergistic effect by the lower CI value. Overexpression of HSP 105 could enhance apoptosis via caspase activation, cytochrome c release from mitochondria, and/or via activation of stress-activated protein kinases, p38 as well as the c-Jun NH2-terminal kinases (JNK) pathways [27]. Combinatorial treatment of ES60 + TC3 served as a better combination to increase HSP 105 expression.

Upon activation by environmental stress, JNK can phosphorylate and promote transcription of proteins in the AP-1 transcription factor complex, including JunB, JunD, ATF2, and c-Jun [28]. c-Jun is a proto-oncogene that can promote formation and growth of breast cancer tumor in nude mice and overexpression of the gene may reduce sensitization of MCF-7 to tamoxifen [29]. c-Jun mRNA expressions were elevated after treatment with TC3 and TC6, while coupling of the drug to *E. scaber* greatly reduced the expression of this gene (Figure 9). Estrogen was found to increase c-Jun expression and tamoxifen decreased it in MCF-7 cells previously [30]; however, in another study by Schiff et al., MCF-7 tumors that exhibited tamoxifen-resistant phenotype expressed more c-Jun resulting from tamoxifen-induced oxidative stress [31]. This explains stimulatory effect by low concentrations of tamoxifen on c-Jun expression, and synergism between *E. scaber* and tamoxifen was able to prevent MCTS growth by downregulation of c-Jun. It is postulated that *E. scaber* extract might have supported tamoxifen in its action and reduced drug resistance as treatment with ES60 + TC6 showed lower c-Jun expression than ES60 + TC3. Absence of c-Jun was shown to augment the expression of p53 and its downstream target p21^Cip1^ in cell cycle regulation [32]. Therefore, it is postulated that downregulation of c-Jun by ES60, either alone or in combination with tamoxifen, might increase amount of p53 and p21^Cip1^ proteins in the MCTS cultures, this leads to cell cycle arrest and apoptosis. This postulate is believed to be true as our previous study found increased expression of p53 protein in MCF-7 monolayer cells treated with *E. scaber* ethanol extract [14].

VEGF is an angiogenic factor that stimulates proliferation and neovascularization of MCF-7 breast tumors [33]. VEGF stimulates the expression of ICAM1, which promotes metastatic ability of MCF-7 cell lines *in vitro* [34, 35]. In this study, expressions of both ICAM1 (Figure 11) and VEGF (Figure 12) were upregulated with increasing dosage of tamoxifen, while treatment by *E. scaber* and the herb-drug combinations was able to downregulate the expression of both genes. Decreased VEGF promotes cell death by preventing phosphorylation of Akt and subsequently downregulates ICAM1 [36]. Tamoxifen was found to decrease VEGF expression; however, breast cancer cells that have *de novo* resistance or acquired resistance towards tamoxifen treatment showed upregulated VEGF expression, and this has been demonstrated in MCF-7 cells previously [33–35]. This explains that our treated cells have developed resistance towards tamoxifen at higher concentration. Combination treatment helped to overcome this treatment resistance and kept the VEGF and ICAM expression lower than control and tamoxifen single treatment to promote more cell death. Growth inhibitory effect by *E. scaber*, either alone or in combination with tamoxifen, could be modulated via its ability to inhibit the prosurvival VEGF and ICAM1 gene expression.

Our previous monolayer breast cancer cells study showed that ethanol extract of *E. scaber* inhibited cell growth and caused MCF-7 cell death via p53-dependent apoptosis [14]. A few compounds isolated from *E. scaber* also showed significant cytotoxicity and antiproliferation activities on MCF-7 cells: Lupeol (a triterpeniod) induced MCF-7 cell apoptosis via downregulated Bcl-2 and Bcl-xL protein expressions [37], scabertopinolide G exhibited strongest cytotoxity towards MCF-7 among all the other 7 germacranolides [38], and deoxyelephantopin (a germacranolide sesquiterpene lactone) induced apoptosis in MCF-7 and mammary adenocarcinoma TS/A cells [39]. It is worth noting that various active compounds in our *E.* scaber ethanol extract may react synergistically or conflicting with each other in certain cellular or protein activity, suggesting specific study of active compound with tamoxifen treatment in future. In overall, our study has complemented the current findings to introduce *E. scaber* extract as an effective medicinal herb to be added with tamoxifen treatment for estrogen receptor-positive breast cancer.

## 5. Conclusions

Combinatorial treatment of *E. scaber* ethanol extract and tamoxifen (with concentrations lower than their respective IC_50_ values on MCTS) had successfully induced greater apoptosis in the cultures of MCF-7 compared to their individual treatment. The treated MCTS showed lower mitochondrial activity, cellular membrane damage, and higher depolarization of mitochondrial membrane potential. The treated MCTS also experienced cellular DNA fragmentation and the S phase cell cycle arrest, which inevitably contributed to cell death. Flow cytometric analysis of externalization of phospatidylserine and acridine orange/propidium iodide staining confirmed that the cell death was mainly due to apoptosis. Further exploration showed that herb-drug treatment elevated caspases-8 and -9 activities but not significant (*p* > 0.05). The treatment was able to upregulate the expression of HSP 105 and downregulate the expression of prosurvival genes such as c-Jun, ICAM1, and VEGF (*p* < 0.05), which favour the cell death of MCTS by the combination treatment. This study reported novel synergism between *E. scaber* and tamoxifen using MCTS, which represents high resemblance to a 3-dimensional tumor. The coupling of *E. scaber* to low concentrations of the drug may provide a better cytotoxic effect against solid tumor of estrogen receptor-positive breast cancer by negating drug resistance. Future investigation may study closely the global transcriptome analysis to provide an overview of the mechanisms regulated by the combination since the specific regulation of caspase-independent apoptosis was recorded in the specific gene expression study for the MCTS generated using more of the breast cancer cell lines treated with the combination. Besides, previously identified active compounds by *E. scaber* such as deoxyelephantopin [13] and lupeol [37] that interacted with tamoxifen shall be performed to support the use of *E. scaber* as a complementary medicine for breast cancer.

## Figures and Tables

**Figure 1:** Representative MTT assay showing the interaction between various combinations of *E. scaber* ethanol extract (ES) and tamoxifen citrate (TC) in MCF-7 multicellular tumor spheroidal (MCTS) cultures after 4 days of incubation *in vitro*. The concentrations of *E. scaber* are indicated on the *χ*-axis, while each line represents viability of cells after treatment by *E. scaber* alone (×) or by 1.56 *μ*g/mL (▲), 3.125 *μ*g/mL (■), or 6.25 *μ*g/mL (♦) of tamoxifen in combination with increasing concentrations of the extract. Cell viability was determined by comparing to the survival of cells in the untreated (negative control) cultures, which was normalized to 100%. The results are presented as means ± SEM from three independent replicates.

**Figure 2:** Cytotoxicity of MCF-7 spheroid cultures towards *E. scaber* ethanol extract 60 *μ*g/mL (ES60), tamoxifen citrate 3.125 *μ*g/mL (TC3), tamoxifen citrate 6.25 *μ*g/mL (TC6), and their combinatorial treatment after 4 days of treatment. Cytotoxicity was evaluated by measuring LDH release into the media in comparison to the maximum LDH release. The results are presented as means ± SEM of three independent experiments. ∗Statistical significance (*p* < 0.05) between control cells and treatment groups.

**Figure 3:** Flow cytometric analysis of phosphatidylserine externalization on MCTS culture after 4 days of treatment. *E. scaber* ethanol extract 60 *μ*g/mL (ES60), tamoxifen citrate 3.125 *μ*g/mL (TC3), and tamoxifen citrate 6.25 *μ*g/mL (TC6). The results are presented as means ± SEM of three independent experiments. Viable—AnnV−/PI−; early apoptosis—AnnV+/PI−; late apoptosis—AnnV+/PI+; dead—AnnV−/PI+; AnnV represents annexin V, PI represents propidium iodide, and +/− represents positive/negative observation of the staining. ∗Statistical significance (*p* < 0.05) between control cells and treatment groups.

**Figure 4:** Fluorescent microscopy observation of apoptosis in MCTS cultures of MCF-7 after dual staining with acridine orange and propidium iodide. The cultures were incubated for 4 days (a) without treatment or with treatment of (b) *E. scaber* ethanol extract 60 *μ*g/mL (ES60), (c) tamoxifen citrate 3.125 *μ*g/mL (TC3), (d) tamoxifen citrate 6.25 *μ*g/mL (TC6), (e) ES60 + TC3, (f) ES60 + TC6 before subjected to acridine orange and propidium iodide staining.

**Figure 5:** Cell cycle distribution of viable MCTS cells in the G0/G1, G2 + M, and S phases of cell cycle. Flow cytometric cell cycle analysis was carried out after 4 days of treatment with *E. scaber*, tamoxifen citrate, and their combinatorial treatment. The population of dead cells in subG0/G1 was ignored in the calculation, and the percentage distribution of the nondead cells was adjusted to 100%. Recalculated percentages of the cells in each phase are presented as means ± SEM of three independent experiments: *E. scaber* ethanol extract 60 *μ*g/mL (ES60), tamoxifen citrate 3.125 *μ*g/mL (TC3), and tamoxifen citrate 6.25 *μ*g/mL (TC6). ∗ Statistical significance (*p* < 0.05) between control cells and treatment groups.

**Figure 6:** Changes of mitochondrial membrane potential (ΔΨm) in MCTS cultures after incubation for 4 days (a) without treatment or with treatment of, (b) *E. scaber* ethanol extract 60 *μ*g/mL (ES60), (c) tamoxifen citrate 3.125 *μ*g/mL (TC3), (d) tamoxifen citrate 6.25 *μ*g/mL (TC6), (e) ES60 + TC3, (f) ES60 + TC6. The results are expressed as fold change relative to Ψm of the untreated control group. The results are presented as means ± SEM of three independent experiments. ∗Statistical significance (*p* < 0.05) between control cells and treatment groups.

**Figure 7:** Effects of *E. scaber*, tamoxifen citrate, and their combinatorial treatment on DNA fragmentation of MCTS cultures. *E. scaber* ethanol extract 60 *μ*g/mL (ES60), tamoxifen citrate 3.125 *μ*g/mL (TC3), and tamoxifen citrate 6.25 *μ*g/mL (TC6). The results are expressed as percentage of cells that was stained by terminal dUTP nick-end labelling (TUNEL positive). Data are presented as means ± SEM of three independent experiments. ∗Statistical significance (*p* < 0.05) between control cells and treatment groups.

**Figure 8:** Caspase-8 and caspase-9 activities of MCF-7 cells in MCTS cultures after 4 days of treatment with *E. scaber*, tamoxifen citrate, and their combinatorial treatment. *E. scaber* ethanol extract 60 *μ*g/mL (ES60), tamoxifen citrate 3.125 *μ*g/mL (TC3), and tamoxifen citrate 6.25 *μ*g/mL (TC6). The results are expressed as fold change relative to the untreated control group. Data are presented as means ± SEM of three independent experiments. ∗Statistical significance (*p* < 0.05) between control cells and treatment groups.

**Figure 9:** Gene expression of c-Jun in MCTS cultures treated by *E. scaber*, tamoxifen citrate, and their combinatorial treatment as measured by real-time quantitative PCR. *E. scaber* ethanol extract 60 *μ*g/mL (ES60), tamoxifen citrate 3.125 *μ*g/mL (TC3), and tamoxifen citrate 6.25 *μ*g/mL (TC6). The results are expressed as fold change relative to the untreated control group. Data are presented as means ± SEM of three independent experiments. ∗Statistical significance (*p* < 0.05) between control cells and treatment groups.

**Figure 10:** Gene expression of heat shock protein (HSP 105) in MCTS cultures treated by *E. scaber*, tamoxifen citrate, and their combinatorial treatment as measured by real-time quantitative PCR. *E. scaber* ethanol extract 60 *μ*g/mL (ES60), tamoxifen citrate 3.125 *μ*g/mL (TC3), and tamoxifen citrate 6.25 *μ*g/mL (TC6). The results are expressed as fold change relative to the untreated control group. Data are presented as means ± SEM of three independent experiments. ∗Statistical significance (*p* < 0.05) between control cells and treatment groups.

**Figure 11:** ICAM1 gene expression in MCTS cultures treated by *E. scaber*, tamoxifen citrate, and their combinatorial treatment as measured by real-time quantitative PCR. *E. scaber* ethanol extract 60 *μ*g/mL (ES60), tamoxifen citrate 3.125 *μ*g/mL (TC3), and tamoxifen citrate 6.25 *μ*g/mL (TC6). The results are expressed as fold change relative to the untreated control group. Data are presented as means ± SEM of three independent experiments. ∗Statistical significance (*p* < 0.05) between control cells and treatment groups.

**Figure 12:** Gene expression of VEGF-A in MCTS cultures treated by *E. scaber*, tamoxifen citrate, and their combinatorial treatment as measured by real-time quantitative PCR. *E. scaber* ethanol extract 60 *μ*g/mL (ES60), tamoxifen citrate 3.125 *μ*g/mL (TC3), and tamoxifen citrate 6.25 *μ*g/mL (TC6). The results are expressed as fold change relative to the untreated control group. Data are presented as means ± SEM of three independent experiments. ∗Statistical significance (*p* < 0.05) between control cells and treatment groups.

**Table 1:** Sequence and properties of genes designed for real-time PCR gene expression study.

Gene		Primer sequence (5′–3′)	Tm (°C)	Product size (bp)	Accession no.
GAPDH	*F*	GGATTTGGTCGTATTGGGC	60.15	206	NM_002046.3
	*R*	TGGAAGATGGTGATGGGATT	60.13		
18S rRNA	*F*	GATGCGGCGGCGTTATTC	58.50	120	X03205.1
	*R*	GTGGTGCCCTTCCGTCAA	56.20		
*β*-actin	*F*	CCATCGTCCACCGCAAAT	57.34	308	NM_001101.3
	*R*	GACTTCCTGTAACAACGCATCT	58.85		
c-Jun	*F*	CGACCTTCTATGACGATGCC	57.90	239	NM_002228.3
	*R*	CCCGTTGCTGGACTGGA	57.50		
HSP 105	*F*	AGATGAAGCAGTAGCCAGAG	54.84	392	AF161368.1
	*R*	CCACCATAGATGCCGTAG	54.89		
ICAM 1	*F*	GACCCCAACCCTTGATGATA	59.61	265	NM_000201.2
	*R*	GTGCTTTTGTGCCGATAGAA	58.92		
VEGF	*F*	GCTGTGGACTTGAGTTGGG	55.60	195	NM_001204385.1
	*R*	GCTGGGTTTGTCGGTGTT	55.90		

∗Tm—melting temperature, *F—*forward primer, *R—*reverse primer.

## Data Availability

The data used to support the findings of this study are included within the article.
